# Identification of 9 Gene Signatures by WGCNA to Predict Prognosis for Colon Adenocarcinoma

This article has been retracted.

**DOI:** 10.1155/2022/8598046

**Published:** 2022-03-29

**Authors:** Mian Yang, Haibin He, Tao Peng, Yi Lu, Jiazi Yu

**Affiliations:** ^1^Department of Colon Anorectal Surgery, Lihuili Hospital, Ningbo Medical Center, Ningbo, Zhejiang, China; ^2^Department of Gastrointestinal Surgery, Lihuili Hospital, Ningbo Medical Center, Ningbo, Zhejiang, China; ^3^Department of Chemoradiotherapy, Lihuili Hospital, Ningbo Medical Center, Ningbo, Zhejiang, China

## Abstract

**Background:**

A risk assessment model for prognostic prediction of colon adenocarcinoma (COAD) was established based on weighted gene co-expression network analysis (WGCNA).

**Methods:**

From the Cancer Genome Atlas (TCGA) database, RNA-seq data and clinical data of COAD patients were retrieved. After screening of differentially expressed genes (DEGs), WGCNA was performed to identify gene modules and screen those associated with COAD progression. Then, via protein-protein interaction (PPI) network construction of module genes, hub genes were obtained, which were then subjected to the least absolute shrinkage and selection operator (LASSO) and Cox regression to build a hub gene-based prognostic scoring model. The receiver operating characteristic curve (ROC curve) was plotted for the optimal cutoff (OCO) of the risk score, based on which, patients were assigned to high or low-risk groups. Areas under the ROC curve (AUCs) were calculated, and model performance was visualized using Kaplan–Meier (KM) survival curves and verified in the external dataset GSE29621. Finally, the model's independent prognostic value was evaluated by univariate and multivariate Cox regression analyses, and a nomogram was built.

**Results:**

Totally 2840 DEGs were screened from COAD dataset of TCGA, including 1401 upregulated ones and 1439 downregulated ones, which were divided into 10 modules by WGCNA. The eigenvalue of the black module was found to have a high correlation with COAD progression. PPI interaction networks were constructed for genes in the black module, and 34 hub genes were obtained by using the MCODE plug-in. A LASSO-Cox regression approach was utilized to analyze the hub genes, and a prognostic risk score model based on the signatures of 9 genes (CHEK1, DEPDC1B, FANCI, MCM10, NCAPG, PARPBP, PLK4, RAD51AP1, and RFC4) was constructed. KM analysis identified shorter overall lower survival in the high-risk group. The model was verified to have favorable predictive ability through training set and validation set. The nomogram, composed of tumor node metastasis (TNM) staging and risk score, was of good predictability.

**Conclusions:**

The COAD prognostic risk model constructed upon the signatures of 9 genes (CHEK1, DEPDC1B, FANCI, MCM10, NCAPG, PARPBP, PLK4, RAD51AP1, and RFC4) can effectively predict the survival status of COAD patients.

## 1. Introduction

Global cancer statistics in 2020 showed that colon cancer (CC) ranked fifth in incidence and mortality among all cancers worldwide, with nearly 1.148 million new cases and 578,000 deaths, accounting for approximately 6.0% of all new cases and deaths of malignancies [1]. CC is highly heterogeneous, and even tumors of the same type with similar characteristics will exhibit different biological behaviors [2]. With adverse prognosis, colon adenocarcinoma (COAD) is the most prevalent one among all kinds of histologic types, occurring primarily in the intestinal mucosa and usually growing in the intestinal lumen and spreading to adjacent organs [3]. Its mortality and recurrence are high, as it is a highly aggressive malignancy [4]. There is a strong connection between the prognosis of COAD and the diagnostic stage. Through early screening and effective treatment, the five-year survival rate can reach 90%. However, because the early symptoms are not obvious, some patients developed metastasis at the initial diagnosis, so much so that even when they receive systemic treatment, the 5-year relative survival is only 14% [5]. Besides, TNM staging, as an extensively applied prognosis evaluation tool based primarily on clinical presentations, cannot reveal its biological heterogeneity [6]. Clinically, accurate prediction of COAD patients' survival can help clinical individual decision making. Therefore, there is an urgent need for more accurate predictive tools that can combine clinical, pathological, and molecular features.

Today, the rapid development of whole genome sequencing technology in the era of precision medicine and the emergence of various bioinformatics analysis tools and public databases make it more convenient to identify key genes from high-throughput data [7]. Therefore, distinguishing individual differences from genetic and molecular level is a vital approach to improve the diagnosis, treatment, and prognosis evaluation system of CC. The gene expression value of tumor is defined by objective value, which avoids subjective bias [8]. Through bioinformatics, multiple biomarkers and risk prediction models that can be used as prognosis prediction of COAD have been identified in recent years. For example, Dong et al. [9] found that MYC and KLK6 can be candidate prognostic predictors and therapeutic targets for COAD patients. In addition, Zhu et al. [10] constructed a COAD risk prediction model and a nomogram that were able to predict patients' overall survival (OS).

The metabolic network, protein interaction network, signal transduction network, and gene expression network that exist in the biological environment all perform their functions in a scale-free (SF) topological distribution [11]. Genes are gathered in the form of co-expression network, in which the ones connected with more genes are in the core position in modules with high modular identity, which are called hub genes [12]. As a potent tool to search for highly correlated gene modules, weighted gene co-expression network analysis (WGCNA) explores the correlation of gene modules with clinical features of interest by means of gene co-expression networks (GCNs) and screens out hub genes within the network [13]. Herein, after retrieving RNA-seq data and clinical baseline data of COAD patients from public databases, co-expression networks were established to mine modules associated with COAD development. In addition, the candidate genes were studied in depth and bioinformatics analysis was combined to build a COAD risk assessment model to verify its prognostic value, providing reference for clinical treatment of COAD patients as well as prognosis improvement.

The rest of the paper is organized as follows.  Section 2 presents the methods. Results are discussed in Section 3. A detailed discussion on the results is made in Section 4, and the paper is concluded in Section 5.

## 2. Methods

### 2.1. Data Source

From the Cancer Genome Atlas, the RNA-seq data and COAD patients' clinical baseline data were retrieved, including 471 cancer samples and 41 adjacent normal counterparts. Then, based on the data integrity of clinical sample information and the matching degree with the sequenced samples, screening was performed to eliminate duplicated and censored data and cases with missing clinical consequences. When different probes corresponded to the same gene name, the mean was taken for subsequent analysis, and low-expression genes (genes with 0 FPKM expression in 50% or more samples) were eliminated to ensure sufficient expression of the genes included in the analysis. In addition, from the GEO database, we chose the GSE29621 dataset [14] that included 65 CC cases and their clinical information. In our research, TCGA-COAD and GSE29621 were used as training set and validation set, respectively.

### 2.2. Differentially Expressed Gene (DEG) Screening

The limma package (v3.40.2) of the R software was utilized to screen DEGs in COAD under the conditions of |logFC| ≧ 1 and adjusted *P* < 0.05. DEG heat maps and volcano plots were created using pheatmap package and ggplot2, respectively.

### 2.3. Weighted Gene Co-Expression Network Analysis (WGCNA)

Using the WGCNA package of R, the DEGs were included in WGCNA to calculate the Pearson correlation coefficient between genes, and a feasible soft threshold *β* was chosen for ensuring SF network. The gene network was constructed by the one-step method. After transforming the adjacency matrix into a topological overlap matrix (TOM), a hierarchical cluster tree of genes was generated by hierarchical clustering. The identification of highly correlated co-expressed gene modules was made by the dynamic tree cut method, and the connection between the module eigengene (ME) and clinical features was analyzed using the Pearson correlation coefficient.

### 2.4. Protein-Protein Interaction (PPI) Network Construction and Hub Gene Screening

Identification of known proteins and PPI prediction were carried out by the STRING database (https://string-db.org/). The PPI networks were evaluated and visualized by Cytoscape (v3.8.2), and the included hub genes were further screened by Molecular Complex Detection (MCODE) in the software with the screening criteria listed in Table 1. Degree cutoff = 2, node density cutoff = 0.1, node score cutoff = 0.2, *κ*-core = 2, and max.depth = 100.

### 2.5. Functional Enrichment Analysis

Gene ontology (GO) analysis was made using the DAVID database, and the functional enrichment of gene sets was analyzed through the DAVID online tool, with *P* < 0.05 as the screening standard.

### 2.6. LASSO Model Building

After feature selection by LASSO regression algorithm, 10-fold cross-validation was adopted to determine parameters to get an appropriate model. Then, the obtained genes were included in the multivariate Cox regression to calculate their regression coefficients, so as to construct the risk scoring equation. After assigning the patients into high and low-risk groups based on the optimal cutoff (OCO), Kaplan–Meier (KM) survival analysis was performed to compare the OS, and time-dependent ROC was utilized for predictive value assessment of gene markers.

### 2.7. Cox Univariate and Multivariate Regression Analyses

With Statistical Package for the Social Sciences (SPSS) 22.0, Cox regression analysis was carried out, and the *P* value, HR, and 95% confidence interval (CI) of each variable were reported by drawing forest plots by GraphpadPrism 8.0. On the basis of multivariate Cox proportional hazard model, a nomogram was built with RMS package for predicting patients' 1, 3, and 5-year survival.

### 2.8. KM Survival Analysis

Survival analysis using Survival in the R package is as follows: P-values and hazard ratios (HRs) with 95% confidence intervals (CIs) in Kaplan–Meier curves were derived by logrank tests and univariate Cox proportional hazards regression.

### 2.9. Statistical Processing

DEG analysis adopted the unpaired Wilcox test, and the *P* value in DEG and enrichment analyses was corrected by the Benjamini and Hochberg approach [15] for false discovery rate (FDR). FDR is a way of understanding the rate of mistakes in null hypothesis testing, in multiple comparisons.

All statistical analyses were realized by R software (v3.40.2) and SPSS 22.0. Except for DEG and enrichment analyses, differences with two-tailed *P* < 0.05 were deemed significant.

## 3. Results

### 3.1. DEG Identification in TCGA-COAD

A total of 471 COAD samples and 41 normal counterparts were obtained from TCGA-COAD, which were displayed by plotting a heat map according to the gene expression in each sample (Figure 1(a)). Totally 1401 overexpressed genes and 1439 underexpressed ones were sorted out, as depicted in Figure 1(b).

### 3.2. Co-Expression Network Construction and Gene Module Identification

The abnormal outliers in TCGA database were removed, and then network building and module clustering were carried out step by step. In order to construct a SF GCN, Pearson correlation matrix computing of all gene pairs was conducted first, followed by weighted adjacency matrix construction. The selection of the optimal soft threshold *β* should satisfy that the constructed GCN approximates a SF topology distribution, that is, the minimum soft threshold when the fitting coefficient R2 approaches or reaches 0.9. As shown in Figures 2(a) and 2(b), when we choose *β* = 7 as the soft threshold of this study, its fitting coefficient *R*^2^ = 0.90, which conforms to the SF topological distribution.  Figure 2(c) shows a gene cluster tree based on hierarchical clustering analysis of adjacency value difference. This study identified 10 modules, and their correlations with clinical features and *P* value calculation were performed by Pearson correlation analysis. The ME of the black module was found to have a strong connection with tumor progression, as shown in Figure 2(d).  Figure 2(e) shows the correlation between GS values of tumor progression traits and MM values of the black module, which can be seen as highly correlated.

### 3.3. PPI Network Construction and Hub Gene Selection

The 71 genes found in the black module, consisting of 71 nodes and 831 edges, were introduced into the STRING to obtain the preliminary PPI network. Using the MCODE plug-in of the Cytoscape, the most important module within the obtained PPI network was found, which consisted of 34 nodes and 507 edges. The visualization results are shown in Figure 3(a), and the yellow module is the most important module. GO functional enrichment analysis of these 34 genes showed the dominant enrichment of these genes in the mitotic cell cycle process and the cell cycle, as illustrated in Figure 3(b).

### 3.4. LASSO Regression and Risk Prediction Model Construction and Verification

Based on the minimum criterion (Lambda.min = 0.0146), 9 genes (CHEK1, DEPDC1B, FANCI, MCM10, NCAPG, PARPBP, PLK4, RAD51AP1, and RFC4) that can effectively predict the prognosis of COAD were obtained by further dimensionality reduction of 34 genes via LASSO regression, as shown in Figure 4(a), and a prediction model based on the signatures of the 9 genes was constructed, as presented in Figure 4(b).

(1) $$\begin{array}{c} \text{Risk score}=\left(-0.0183\right)*\text{CHEK}1+\left(-0.096\right)*\text{DEPDC}1\text{B}+\left(0.2645\right)*\text{FANCI}\\ +\left(0.2622\right)*\text{MCM}10+\left(-0.2219\right)*\text{NCAPG}+\left(-0.4163\right)*\text{PARPBP}\\ +\left(-0.5178\right)*\text{PLK}4+\left(0.2412\right)*\text{RAD}51\text{AP}1+\left(0.2507\right)*\text{RFC}4. \end{array}$$

According to the ranking of risk scores, we assigned the samples to high and low-risk groups taking the OCO risk score (−0.0352) as the threshold. KM analysis showed an evidently worse prognosis in high-risk group, as shown in Figure 4(c). ROC curves were applied for the sensitivity and specificity of this risk model for OS prediction. In TCGA training set, the AUCs of this risk model for predicting 1, 3, and 5-year survival were 0.670, 0.660, and 0.710, respectively, indicating high accuracy of this model in predicting COAD patients' OS, as illustrated in Figure 4(d). In addition, GSE29621 was used as the validation set, and the OCO risk score (−0.9750) was used as the threshold to assign the samples in the GSE29621 dataset to high and low-risk groups. KM analysis also identified an obviously worse prognosis in high-risk group, as depicted in Figure 4(e). Through the application of ROC curve to verify this model's sensitivity and specificity for predicting patients' OS, we found that the predictive AUC values of the risk model for 1, 3, and 5-year survival were 0.740, 0.640, and 0.680, respectively, which also showed high accuracy, as shown in Figure 4(f).

Accuracy is calculated as accuracy = (TN + TP)/(TN + TP + FN + FP). Similarly, sensitivity = TP/(TP + FN), while specificity = TN/(TN + FP).

### 3.5. Nomogram-Based Risk Prediction Model Establishment

TNM staging and risk score may independently influence COAD patients' outcomes, as indicated by univariate and multivariate Cox regression analyses, as depicted in Figures 5(a) and 5(b). Next, we established a nomogram, as shown in Figure 5(c), based on TNM staging and risk score. According to the actual situation of each variable of a patient, the corresponding scale was found, and the score of each variable was obtained by projecting the scale (points) upward to the top. The total point was obtained by adding the scores, and the patient's 1, 3, and 5-year OS was obtained by projecting downward according to the total score value. The calibration results showed that compared with the ideal model, the 1, 3, and 5-year OS models have favorable predictability, as illustrated in Figure 5(d).

### 3.6. Gene Expression and Prognostic Value in COAD

The expression levels of CHEK1, DEPDC1B, FANCI, MCM10, NCAPG, PARPBP, PLK4, RAD51AP1, and RFC4 in TCGA-COAD patients were analyzed. All the nine genes were highly expressed in COAD compared with normal counterparts, as shown in Figure 6(a). KM analysis identified that of them, only CHEK1, DEPDC1B, and PLK4 had a connection with patients' OS, as presented in Figures 6(b)–6(j). It is worth mentioning that although CHEK1, DEPDC1B, and PLK4 were upregulated in cancer tissues, low CHEK1, DEPDC1B, and PLK4 levels were strongly linked to adverse prognosis (*P* < 0.05).

## 4. Discussion

COAD is one of the most deadly cancers. For the treatment of CC, some prognostic markers have been found, as well as some models to predict clinical outcomes [16, 17]. However, the search for markers or models that can accurately predict prognosis and provide personalized treatment for patients remains critical. Evidence has indicated that genetic factors and clinicopathological features are involved in carcinogenesis and progression [17]. At the same time, the view that COAD is a molecular heterogeneous disease has been gradually recognized due to the study of numerous multiomics data and its analysis results [10, 19]. While assessing their interactions, many studies have begun to highlight changes in whole genome expression in recent years, as they are related to COAD, so as to draw a molecular map of COAD that is more complete [20–22].

In this research, multiple DEGs were obtained by analyzing COAD dataset in TCGA database, and then the gene modules related to COAD progression were screened by WGCNA for in-depth study of the module genes. LASSO regression is a penalized regression method that shrinks some coefficients to get a more refined model by constructing a penalty function. It is a biased estimation that deals with data with complex collinearity, which is often used in high-dimensional regression and can make up for the deficiency of univariate Cox regression analysis [23, 24]. After further processing by LASSO regression, 9 genes related to tumor progression were finally obtained, which were then included in the multivariate Cox regression to build a risk model for prognosis prediction. Furthermore, via ROC curve verification of the model performance, it was found that its ability to predict COAD patients' 1, 3, and 5-year survival in the training set and verification set was moderately accurate. Finally, univariate as well as the final multivariate COX regression analysis identified the independence of TNM staging and the risk model as prognostic markers. Based on this model, we constructed a nomogram and found that it was well calibrated. Some previous studies have built risk models that can predict the prognosis of COAD, many of which include multiple functional gene sets. For example, Wang and Liu [25] constructed and verified a CC prognostic risk model based on 5 immune genes. Chen et al. [26] identified a new genetic marker related to COAD invasion. This study not only constructed a risk model for prognosis prediction of COAD but also built a nomogram based on this model to jointly evaluate the prognosis of patients with TNM staging, providing ideas and directions for the basic research of COAD.

The 9 genes identified are CHEK1, DEPDC1B, FANCI, MCM10, NCAPG, PARPBP, PLK4, RAD51AP1, and RFC4, respectively, which all presented upregulated expression in TCGA-COAD patients. However, only three genes were significantly correlated with patient prognosis, namely, CHEK1, DEPDC1B, and PLK4. What is more notable is that downregulation of the three genes was strongly linked to patients' adverse prognosis. Belonging to the CHEK family, CHEK1 is a serine/threonine-specific protein kinase that mediates cell cycle arrest in DNA injury [27]. As an important participator in coordinating DNA repairing, CHEK is an important field of cancer progression and treatment [28]. CHEK1 was considered as a tumor suppressor in the past [29]. Previous studies mostly reported that it was upregulated in multiple cancers, including cervical carcinoma [30], colorectal carcinoma [31], and liver carcinoma [32], while some others showed that it was downregulated in brain cancer and central nervous system cancer [33, 34]. We found that CHEK1 was upregulated in COAD. In addition, it is shown that CHEK1 can be post-transcriptionally modulated by microRNAs—vital regulators of tumor growth and therapeutic response [35]. Thus, the CHEK1 gene may have carcinogenic or anti-cancer properties, which is up to the cancer type. This study also found a connection between low CHEK1 expression in COAD and adverse prognosis of patients, which also agrees with previous research [36]. DEPDC1B was first identified in the mRNA expression profile of human breast cancer MDA-MB231 cells [37]. In mitosis, DEPDC1B is necessary to coordinate death events and cell cycle processes [38]. It has been reported to be upregulated in oral carcinoma [39], non-small-cell lung carcinoma [40], soft tissue sarcoma [41], malignant melanoma, etc. Besides, elevated DEPDC1B is shown to suggest shorter biochemical relapse-free survival in prostate cancer patients [42]. In this study, however, it is the downregulated DEPDC1B that is associated with adverse prognosis. At present, the connection between DEPDC1B and the prognosis of CC has not been well documented, which can be further explored as a breakthrough point in future research. As to PLK4, it is a serine/threonine protein kinase that modulates centriole duplication [43]. Overexpression of PLK4 can give rise to abnormal number of centrosomes, mitotic defects, and chromosome instability, causing tumorigenesis [44]. Therefore, PLK4 has become a therapeutic target for a wide range of tumors. In addition, PLK4 is found in various tumor types and has a close connection with cancer patients' outcomes [45, 46]. For example, via regulating the Wnt/*β*-catenin axis, the elevated PLK4 accelerates colorectal cancer progression and induces epithelial-mesenchymal transition [47], which is similar to our findings, while conversely, PLK4 downregulation suppresses cell apoptosis, and underexpressed PLK4 is linked to unfavorable prognosis of hepatocellular carcinoma [48]. Therefore, the role of PLK4 in COAD warrants further study.

## 5. Conclusion

To sum up, this study used bioinformatics methods such as WGCNA to study the RNA-seq data and COAD patients' clinical data from TCGA database and successfully built a risk model of prognosis prediction based on 9 gene signatures, with good performance, indicating its feasibility as a novel prognostic indicator of COAD. Despite the rigorous screening, this research still has some limitations. First of all, due to the limited length, the specific biological functions of the 9 risk genes need to be further explored, especially the correlation between the expression of CHEK1, DEPDC1B, and PLK4 and the prognosis of COAD patients. Second, although the TCGA database is large in number and scale, it mainly targets the Caucasian population, so the applicability of the model to the yellow race of Asia needs to be verified on a larger scale of data. Overall, this research provides ideas and directions for the basic research of COAD, and we will follow up with more *in vitro* and *in vivo* experiments, as well as clinical samples for further verification and molecular mechanism research.

## Figures and Tables

**Figure 1:** DEG screening. (a) Heat map showing DEGs in TCGA-COAD. (b) Volcano plot showing DEGs in TCGA-COAD (DEG: differentially expressed gene).

**Figure 2:** Co-expression network construction and gene module identification. (a) Fitting coefficient R2 as a function of a soft threshold parameter in the scale-free topology model. (b) Mean connectivity as a function of a soft threshold parameter. (c) Gene cluster tree based on hierarchical clustering analysis of adjacency difference. (d) Heat map of the relationship between gene modules and clinical features. (e) Correlation between gene signatures for tumor and module membership in the black module.

**Figure 3:** PPI network analysis of black module genes. (a) PPI networks and 34 hub genes identified by MCODE plug-in. (b) GO functional enrichment analysis of hub genes (PPI: protein-protein interaction; GO: gene ontology).

**Figure 4:** Prognostic risk model construction and verification. (a) LASSO for risk factor screening. (b) LASSO variable trajectory diagram. (c) KM curves of high and low-risk groups of the risk model constructed by 9 gene signatures (training set). (d) ROC curve validation for the validity of the model (training set). (e) KM curves of the high and low-risk groups (validation set). (f) ROC curve validation for the validity of the model (validation set).

**Figure 5:** Nomogram-based risk prediction model establishment. (a) Forest plot displaying univariate Cox regression analysis of gene signatures. (b) Forest plot displaying multivariate Cox regression analysis of gene signatures. (c) Nomogram-based prognosis prediction model. (d) Calibration curve of the nomogram.

**Figure 6:** Expression of 9 genes and their correlations with patient survival. (a) Expression of 9 genes. (b) KM survival curve of CHEK1 in cases. (c) KM survival curve of DEPDC1B in cases. (d) KM survival curve of FANCI in cases. (e) KM survival curve of MCM10 in cases. (f) KM survival curve of NCAPG in cases. (g) KM survival curve of PARPBP in cases. (h) KM survival curve of PLK4 in cases. (i) KM survival curve of RAD51AP1 in cases. (j) KM survival curve of RFC4 in cases.  ^*∗∗∗*^*P* < 0.0001; KM survival curve: Kaplan–Meier survival curve.

**Table 1:** Screening criteria for MCODE.

Criteria	Number
Degree cutoff	2
Node density cutoff	0.1
Node score cutoff	0.2
*κ*-core	2
Max depth	100z

## Data Availability

Previously reported bioinformatics data were used to support this study and are available at doi.org/10.1007/s11605-011-1815-0. These datasets are cited at relevant places within the text as references [14].
